# miR-139-5p Suppresses Proliferation and Angiogenesis of Intracranial Aneurysm via FGB

**DOI:** 10.1155/2022/5824327

**Published:** 2022-04-16

**Authors:** Tao Jin, Gong Chen, Qingzhu An, Xuanfeng Qin, Yuanyuan Hu, Yan Yan, Jia Hu, Bing Zhou, Bing Leng

**Affiliations:** ^1^Department of Neurosurgery, Huashan Hospital, Fudan University, Shanghai, China; ^2^Department of Interventional and Vascular Surgery, Affiliated Tenth People's Hospital of Tongji University, Shanghai, China

## Abstract

Intracranial aneurysm (IA) is a common cerebrovascular disease. Understanding the mechanism regulating the progression of IA could help to develop novel therapeutic methods for this disease. In this study, we confirmed FGB is one of the targets of miR-139-5p. Moreover, miR-139-5p expression in intracranial aneurysm specimens was suppressed compared with normal tissues. However, we found that FGB in intracranial aneurysm samples was remarkedly enhanced compared to normal tissues. Moreover, we found miR-139-5p overexpression and FGB silencing inhibit HBMEC proliferation and tube formation and suppressed *α*-SMA and CXCR4 levels in HBMEC cells. Furthermore, a rescue experiment confirmed miR-139-5p affected the proliferation and angiogenesis of HBMEC through FGB. Despite further research being needed to determine the exact functions of miR-139-5p in the formation of CA, our new findings contribute to a comprehensive understanding of the treatment mechanism of IA.

## 1. Introduction

Intracranial aneurysm (IA) is a common cerebrovascular disease [1]. It has high morbidity and mortality in patients aged 40–60 years [1]. It is characterized by abnormal swelling of cerebral arteries [2]. The occurrence of IA may be related to the interruption of normal protein translation in vascular cells [2]. Because of the serious complications caused by these lesions, people are more and more interested in understanding their pathophysiology [3].

MicroRNA is a small noncoding RNA with a length of about 22 nucleotides, and it is an important regulator of various biological processes [4]. Currently, there is evidence that there is a biological link between miRNA and IA. For instance, miR-34a modulates phenotypic modulation of VSM cells via CXCR3 and MMP-2 in IA [5]. miR-21 participated in the formation of intracranial aneurysm through JNK signaling [6]. In recent studies of miRNA and abdominal aortic aneurysm (AAA), the increased expression of miR-21 may be an endogenous response to pathological aortic dilation [7]. Increased expression of miR-21 leads to proproliferation and antiapoptotic responses of VSM cells in the blood vessel wall [7], most likely to protect the aorta from further dilation and eventual rupture [8].

Emerging studies had reported the important regulatory roles of MiR-139-5p in cardiovascular disease (CVD). For example, miR-139-5p was identified as one of the most suppressed miRNAs in the heart of patients with hypertrophic cardiomyopathy (HCM) [9]. This study emphasizes that miR-139-5p is a new antihypertrophic miRNA in cardiomyocytes. miR-139-5p may reduce myocardial hypertrophy by regulating myocardial hypertrophy in vitro. These findings indicate that the miR-139-5p/c-Jun axis is a new target for the prevention and treatment of cardiac remodeling. Moreover, miR-139-5p was identified as a suppressor of myogenesis via suppressing the Wnt/*β*-catenin axis [10]. However, the mechanism and functional roles of miR-139-5p in IA remained to be largely unclear.

Studying miR-139-5p helps to better understand the mechanism of IA. This study focuses on the role of these miR-139-5p in the pathogenesis of IA to further detect the possible targets of miRNA and to further prove their exact role in the pathogenesis of IA.

## 2. Materials and Methods

### 2.1. Cell Culture

Unless otherwise stated, the reagents used in this study were obtained from Millipore Sigma, Burlington, Massachusetts, USA. Human brain microvascular endothelial cells (HBMECs) were obtained from Neuromics (Minneapolis, Minnesota, USA) and cultured at 37°C with 5% CO_2_.

### 2.2. Quantitative PCR (qPCR)

TRIzol was applied to extract RNA based on a previous report [11]. RevertAid first-strand cDNA kit (Waltham Thermal Sciences, Massachusetts, USA) was used to perform RT-PCR to generate complementary DNA (cDNA). Then, PowerTrack SYBR Green Master Mix and related primer pairs were used for qPCR assays. The cycle threshold (Ct) was obtained from three biological replicates, standardized to GAPDH or U6 level, and compared to the control. The relative gene expression was analyzed with the 2^−ΔΔCt^ method [12]. The oligonucleotide sequence is as following: human miR-139-5p (forward) 5′-TGGAGACGCGGCCCTGTT-3′ and (reverse) 5′-TCTACAGTGCACGTGTCT-3′; U6 (forward): 5′-CTCGCTTCGGCAGCACA-3′ and (reverse): 5′-ACGCTTCACGAATTTGCGT-3′; FGB (forward): 5′-AGTGATTCAGAACCGTCAAGAC-3′ and (reverse): CATCCTGGTAAGCTGGCTAATTT-3′; GAPDH (forward): 5′-GGTCTCCTCTGACTTCAACA-3′ and (reverse): GTGAGGGTCTCTCTCTTCCT-3′;

### 2.3. Luciferase Reporter Analysis

To evaluate the effect of miR-139-5p on FGB expression, we transfected a plasmid containing predicted miRNA interaction sites (wild type and mutant) in hBMECs cells using liposomal amine RNAiMAX (Thermo Fisher Scientific). Two days after transfection, the luciferase reporter analysis system (Promega, USA) was used to measure Renilla luciferase activity by normalizing it to firefly luciferase activity.

### 2.4. Western Blot

The western blot was applied as described above, and the Odyssey system was used for verification (LI-COR Biosciences, Lincoln, Northeast, USA). Fiji software was used to quantify the band intensity. The following antibodies were used: FGB (catalogue # ab208247, Abcam, USA); *β*-actin (category number ab8229, Cambridge, Massachusetts, USA); *α*-SMA (Dako GmbH, Germany); and rabbit anti-human CXCR4 (sc-9046, Santa Cruz, CA).

### 2.5. Tube Formation Assay

50 *μ*L growth factor reduced matrix gel (Becton Dickinson) was inoculated on a 96-well plate at 37°C for 30 minutes. Then, 10000 cells were seeded in each well for 3 days. The tube formation rate was analyzed based on Quantity One software (Bio-Rad, Hercules, California, USA).

### 2.6. Cell Proliferation Test

CCK-8 (Dojindo) was applied to detect cell proliferation. In short, the 5000 transfected cells per well are seeded in a 96-well plate, and 10 *μ*L CCK-8 is added to each well at 0, 1, 2, and 3 days after treatment. The OD 450 nm was detected using a microplate reader ELx808 (BioTek).

### 2.7. Tissue Samples

A total of 10 IA samples and 10 control samples were obtained from our hospital. The study was approved by the research ethics committee of our hospital. Informed consent was provided by all patients.

### 2.8. Statistical Analysis

GraphPad 8 (Prism, USA) was used to perform statistical analysis. *p* < 0.05 was regarded as statistical significance. Statistical comparisons were performed using *t*-tests or Mann–Whitney *U*-tests according to the test conditions.

## 3. Results

### 3.1. FGB is the Molecular Target of miR-139-5p

Bioinformatics analysis shows hsa-miR-139-5p is a highly conserved miRNA, which may inhibit the expression of FGB mRNA (Figure 1(a)). Our previous studies found that FGB was significantly upregulated in the intracranial aneurysm group and ruptured aneurysm group by mass spectrometry analysis (data not shown). Here, we speculated that miR-139-5p could target and inhibit FGB expression and improve aneurysm progression. Then, the dual-luciferase reporter assay revealed miR-139-5p mimics remarkedly inhibited the luciferase activities of hBMECs transfected with wildtype 3′-UTR of FGB, not mutated 3′-UTR of FGB (Figure 1(b)).

miR-139-5p was suppressed and FGB was upregulated in intracranial aneurysm samples. To determine whether miR-139-5p and FGB were expressed in intracranial aneurysm tissue, its expression in control tissue and intracranial aneurysm tissue was evaluated by RT-PCR. Compared with control samples, miR-139-5p expression in intracranial aneurysm specimens was significantly downregulated (Figure 1(c)). However, we found that FGB in intracranial aneurysm samples was overexpressed compared to normal samples (Figure 1(d)). Of note, the ELISA assay showed TNF-*α* and LI-1*β* were upregulated in intracranial aneurysm samples (Figures 1(e)–1(f)).

### 3.2. Upregulation of miR-139-5p Inhibits HBMEC Viability and Angiogenesis

To determine whether miR-139-5p can affect HBMEC proliferation and angiogenesis in vitro, we transfected HBMEC with miR-139-5p agomir or antagonist (Figure 2(a)). As shown in Figure 2, miR-139-5p overexpression inhibits HBMEC proliferation and tube formation (Figures 2(b) and 2(c)). On the contrary, suppression of miR-139-5p can enhance HBMEC proliferation and tube formation (Figures 2(b) and 2(c)). *α*-SMA and CXCR4 had been reported to play a crucial role in angiogenesis. Here, we revealed the upregulation and knockdown of miR-139-5p reduced and induced the levels of FGB, *α*-SMA, and CXCR4 in HBMECs by western blot and immunofluorescence staining, respectively (Figures 2(d)–2(g)).

### 3.3. FGB Gene Knockdown Inhibits HBMEC Viability and Angiogenesis

Next, we also detected the role of FGB in HBMEC. As shown in Figure 3, FGB gene knockdown inhibited HBMEC proliferation and tube formation (Figures 3(a) and 3(b)). In contrast, overexpression of FGB enhances the proliferation and tube formation of HBMEC (Figures 3(a) and 3(b)). In addition, we found that FGB knockdown and overexpression significantly reduced and induced the expression of *α*-SMA and CXCR4 in HBMECs, respectively (Figures 3(c)–3(f)).

### 3.4. miR-139-5p Modulated the Proliferation and Angiogenesis of HBMECs through FGB

Furthermore, we conducted rescue experiments to detect whether miR-139-5p modulates the proliferation and angiogenesis of HBMEC through FGB (Figure 4(a)). As shown in Figure 4, our results show that miR-139-5p mock transfection significantly inhibits the proliferation and tube formation of HBMEC, while the cotransfection of FGB overexpression plasmid partially reverses the proliferation and microtubules caused by miR-139-5p inhibition (Figures 4(b) and 4(c)). miR-139-5p mock transfection can significantly reduce the expression of FGB, *α*-SMA, and CXCR4 in HBMEC, and cotransfection with FGB overexpression plasmid can reverse the decrease in FGB, *α*-SMA, and CXCR4 expression induced by miR-139-5p mock transfection (Figures 4(d)–4(g)).

## 4. Discussion

In this study, we reported miR-139-5p in human intracranial aneurysm cells was significantly reduced, which can inhibit the tube-forming ability of HBMECs, while suppressing miR-139-5p can enhance the tube-forming ability of HBMEC. WB and immunofluorescence display miR-139-5p significantly reduced the FGB, *α*-SMA, and CXCR4 expression, and miR-139-5p inhibitor significantly increased the FGB, *α*-SMA, and CXCR4 expression in HBMECs.

Bioinformatics analysis shows that miR-139-5p directly targeted FGB. The dual-luciferase assay confirmed the regulatory relationship between FGB and miR-139-5p. miR-139-5p can target FGB and inhibit FGB expression, thereby improving the progression of aneurysm. FGB was reported to promote smooth muscle and endothelial cell proliferation [13]. Fibrinogen is a biomarker of inflammation, which indicated a high risk of cardiovascular disease [14, 15]. Elevated plasma FGB concentration is usually associated with hypertension and stroke. FGB can raise blood viscosity and peripheral resistance and promote platelet aggregation and endothelial cell development [16]. Therefore, FGB acted as a key regulator of CVD. Other inflammatory biomarkers involved in the synthesis of FGB, such as interleukin (IL)-6 and IL-1, are also associated with increased blood pressure. FGB overproduction and progress are related to high blood pressure and may even be related to the development of hypertension [17]. In the present study, the expression of FGB in the intracranial aneurysm was remarkedly upregulated. Moreover, we observed the levels of IL-1*β* and tumor necrosis factor a (TNF-*α*) increase with the upregulation of FGB in human intracranial aneurysm cells. Interleukin-1 (IL-1) has been reported to play an important role in the immune and inflammatory responses in cerebrovascular diseases [18, 19]. IL-1*β* is one of the 3 members of the IL-1 family, which was highly expressed in intracranial aneurysm samples [20]. Previous studies showed the changes in TNF-*α* are related to human cerebral aneurysms. TNF-*α* participated in modulating multiple proinflammatory genes in cerebral vascular smooth muscle cells, including MMP-3, MMP-9, and IL-1*β* [21]. In this study, we revealed that overexpression of FGB can significantly promote the tube-forming ability of HBMEC, while FGB gene knockdown can inhibit the tube-forming ability of HBMEC. Further experiments showed miR-139-5p transfection can significantly inhibit the tube formation of HBMEC, while cotransfection of FGB overexpression plasmid can reverse the inhibition of miR-139-5p mock transfection on tube formation. In conclusion, our research emphasizes miR-139-5p acted as a new regulator miRNA in IA, which significantly inhibit the tube-forming ability of HBMEC by downregulating FGB in vitro.

However, our research still has many limitations. First, we only verify the data in vitro. The function of miR-139-5p needs to be further verified by in vivo experiments and clinical samples. Therefore, in particular, the predictive performance of these miRNAs may be affected by samples from different sources. Secondly, more detailed mechanisms related studies are still needed to further clarify the effect of miR-139-5p on FGB and FGB's downstream targets. Thirdly, the clinical samples used in this study are limited. Only 10 control and IA samples were included. More validations using a big sample size are still needed.

Overall, our results strongly support the idea that miR-139-5p modulated the pathological process of vascular diseases. Despite further research is needed to determine the exact role of miR-139-5p in the formation of IA, our new findings contribute to a comprehensive understanding of the treatment mechanism of IA.

## Figures and Tables

**Figure 1:** miR-139-5p was suppressed and FGB was upregulated in intracranial aneurysm samples. (a) Schematic illustration indicating the interaction between miR-139-5p and FGB. (b) The dual-luciferase reporter assay revealed miR-139-5p inhibited the luciferase activities of hBMECs transfected with wildtype 3′-UTR of FGB, not mutated 3′-UTR of FGB. (c) miR-139-5p levels in intracranial aneurysm specimens were significantly downregulated. (d) RT-PCR assay showed FGB in intracranial aneurysm samples was induced compared to normal tissues. (e, f) ELISA assay showed TNF-a and IL-1*β* were upregulated in intracranial aneurysm samples.

**Figure 2:** miR-139-5p inhibits HBMEC viability and angiogenesis. (a) The transfection efficacy was determined in HBMECs after transfecting with miR-139-5p agomir or antagonist. (b) The effect of miR-139-5p on HBMEC proliferation. (c) The effect of miR-139-5p on HBMEC tube formation. (d) The levels of FGB, *α*-SMA, and CXCR4 were detected using WB after overexpression and silencing of miR-139-5p in HBMECs. (e–g) The levels of FGB (e), *α*-SMA (f), and CXCR4 (g) were determined using immunofluorescence staining after overexpression and knockdown of miR-139-5p in HBMECs.

**Figure 3:** Knockdown of FGB inhibits HBMEC proliferation and angiogenesis. (a) The transfection efficacy was determined in HBMECs after transfecting with FGB overexpression plasmids and siRNA. (b) The effect of FGB on HBMEC proliferation. (c) The effect of FGB on HBMEC tube formation. (d) The protein levels of FGB, *α*-SMA, and CXCR4 were determined using WB after overexpression and knockdown of FGB in HBMECs. (e–g) The protein levels of FGB (e), *α*-SMA (f), and CXCR4 (g) were determined using immunofluorescence staining after overexpression and knockdown of FGB in HBMECs.

**Figure 4:** miR-139-5p modulated the viability and angiogenesis of HBMEC through FGB. (a) The transfection efficacy was determined in HBMECs. (b, c) The proliferation and tube formation of HBMEC were detected after cotransfection of FGB overexpression plasmid and miR-139-5p. (d) The levels of FGB, *α*-SMA, and CXCR4 were determined using WB after cotransfection of FGB overexpression plasmid and miR-139-5p. (e–g) The levels of FGB (e), *α*-SMA (f), and CXCR4 (g) were determined using immunofluorescence staining after cotransfection of FGB overexpression plasmid and miR-139-5p mimic.

## Data Availability

All the data can be acquired by reasonable request.
